# A Methylation Diagnostic Model Based on Random Forests and Neural Networks for Asthma Identification

**DOI:** 10.1155/2022/2679050

**Published:** 2022-09-28

**Authors:** Dong-Dong Li, Ting Chen, You-Liang Ling, YongAn Jiang, Qiu-Gen Li

**Affiliations:** ^1^Nanchang University, Nanchang, 330006 Jiangxi, China; ^2^Department of Pulmonary and Critical Care Medicine, Jiangxi Provincial People's Hospital, Nanchang, 330006 Jiangxi, China; ^3^Department of Pulmonary and Critical Care Medicine, Wuhan Wuchang Hospital, Wuhan, 430063 Hubei, China

## Abstract

**Background:**

Asthma significantly impacts human life and health as a chronic disease. Traditional treatments for asthma have several limitations. Artificial intelligence aids in cancer treatment and may also accelerate our understanding of asthma mechanisms. We aimed to develop a new clinical diagnosis model for asthma using artificial neural networks (ANN).

**Methods:**

Datasets (GSE85566, GSE40576, and GSE13716) were downloaded from Gene Expression Omnibus (GEO) and identified differentially expressed CpGs (DECs) enriched by Gene Ontology (GO) and Kyoto Encyclopedia of Genes and Genomes (KEGG) analysis. Random forest (RF) and ANN algorithms further identified gene characteristics and built clinical models. In addition, two external validation datasets (GSE40576 and GSE137716) were used to validate the diagnostic ability of the model.

**Results:**

The methylation analysis tool (ChAMP) considered DECs that were up-regulated (*n* =121) and down-regulated (*n* =20). GO results showed enrichment of actin cytoskeleton organization and cell-substrate adhesion, shigellosis, and serotonergic synapses. RF (random forest) analysis identified 10 crucial DECs (cg05075579, cg20434422, cg03907390, cg00712106, cg05696969, cg22862094, cg11733958, cg00328720, and cg13570822). ANN constructed the clinical model according to 10 DECs. In two external validation datasets (GSE40576 and GSE137716), the Area Under Curve (AUC) for GSE137716 was 1.000, and AUC for GSE40576 was 0.950, confirming the reliability of the model.

**Conclusion:**

Our findings provide new methylation markers and clinical diagnostic models for asthma diagnosis and treatment.

## 1. Introduction

Asthma is a chronic, heterogeneous respiratory disease that affects people of all age groups. Recently, asthma-related morbidity and mortality have increased annually. The clinical manifestations of asthma are mainly respiratory symptoms. The main pathological features include chronic airway inflammation, high airway response, and airway remodeling [1–3]. Immunoglobulin E (IgE), interleukin-5 (IL-5) and its receptors, and interleukin-4 (IL-4) receptors are used as molecular targets for clinical diagnosis of asthma; however, specific and individual differences are very large, and the clinical treatment of asthma patients is still inadequate [4, 5].

DNA methylation, a major epigenetic component of humans, has a profound effect on the occurrence and development of various diseases [6, 7]. There is substantial evidence that the mechanisms and characteristics of asthma depend on methylation patterns. Gaffin et al. [8] studied DNA methylation in peripheral blood mononuclear cells nuclear airway epithelial cells of atopic, non-atopic, and healthy asthmatic children and confirmed that multiple CpG sites in the ARDB2 gene promoter region were associated with reduced dyspnea in children. RNA methylation provided new options for asthma treatment [9, 10].

Although multiple studies have been performed to distinguish the disease from healthy patients by identifying CpGs loci, however, the results are not encouraging [11]. Reliable quantitative measurements using fewer markers are a viable option. The application of machine learning technology in the medical field has significantly accelerated the research to understand the diseases [12, 13]. Machine learning can describe the complexity and unpredictability of human diseases as reported in various studies [14–16]. Cao et al. [17] identified key genes for Th2-high asthma using weighted by weighted gene co-expression network analysis. There is currently no standard diagnostic model for screening and early detection of asthma. The rapid development of machine learning methods, such as random forests (RF) and artificial neural networks (ANN), is frequently used in biomarker research [18–21].

This is the first study in which we have analyzed the methylation expression profile of asthma samples by machine learning (RF and ANN) and obtained DECs. The receiver operating characteristic (ROC) curve evaluated the diagnostic performance of our model. The external validation datasets also confirmed the efficiency of the model. This study aimed to identify asthma diseases by analyzing methylation data. The workflow of the study is shown in Figure 1.

## 2. Methods and Materials

### 2.1. Data Acquisition and Preprocessing

The methylation expression profiles GSE85566 [22] (asthma samples: 74, normal samples: 41), GSE40576 [23] (asthma samples: 97, normal samples: 97), and GSE13716 [24] (asthma samples: 16, normal samples: 17) were downloaded from Gene Expression Omnibus (GEO) database. The missing data from expression profiles were filled using the ChAMP package and normalized.

### 2.2. Differential Analysis and Design Grouping of GSE85566 Methylation Expression Profiles

Filter probes (*p*-value < 0.01) through champ.filter function of ChAMP package (version:2.24.0) performed CpGs difference analysis (deltaBeta > 0) with champ function and obtained top 1000 CpGs heat map according to the analysis results of champ. The threshold was deltaBeta <-0.05, *p*-value <-10^−8^, and matched gene symbols based on methylation array 450 k for later GO and KEGG analysis (clusterProfilter, version: 4.3.3). The above analysis was performed using the R environment installation package.

### 2.3. Random Forest (RF) Classification

The DECs obtained by ChAMP were initially identified and classified using the R package randomForest (version 4.7.1). The value of err.rate was minimized by calculating the average model miscalculation rate of all DECs in the data to ensure the best node (mtry). In this study, the optimal variable setting of the binary tree in the node was seven, and the optimal number of trees for the random forest was 600. The Gini coefficient selected significant DECs (top 10) as specific candidates for asthma. The heat map of these DECs was constructed by pheatmap (version: 1.0.12) to show their classification ability.

### 2.4. Artificial Neural Network Model Construction

The artificial neural network model of important candidate variables was constructed using R package (neuralnet, version: 1.44.2). According to the specification, the number of hidden neurons should be 2/3 of the size of the input layer plus 2/3 of the size of the output layer; the number of hidden neurons should be between the sizes of the input layer and output layers. The base expression profile data were normalized (0 to 1) and processed in neuralnet. The output was set to normal and asthma, and the output of the first hidden layer (input of the last output layer) was regarded as the result of gene weights. The termination condition was the absolute derivative of the error function (reaching the threshold < 0.01).

### 2.5. Model Performance Evaluation

Different R packages in the R environment (R version 4.1.3, https://www.r-project.org) were used to evaluate the model performance. For model prediction and identification, caret (version: 6.0-91) and confusionMatrix were used. For RF, pROC (version: 1.18.0) was used, and for ANN and AUC (Area Under Curve), ggplot2 (version: 3.3.5) was used. Classification and Regression Trees (CART), Support Vector Machines (SVM), eXtreme Gradient Boosting (XGBoost) algorithm by rpart (version 4.1.16), xgboost (version 1.6.0.1), and e1071 (version 1.7-9) packages were used for model validation on GSE40576 and GSE137716 datasets.

## 3. Results

### 3.1. CpGs Landscape of GSE85566

Methylation plays a key role in various diseases, as reported previously [25–27]. The methylation ChAMP package champ.DMP was used to analyze and process the methylation expression profile in the dataset GSE85566 (74 asthma samples and 41 normal samples) to understand the methylation structure of asthma samples and to calculate the differential CpGs sites. The top 1000 CpGs heat map landscape (asthma and normal samples) is displayed in Figure 2(a). Further methylation targets were searched to differentiate between asthma and healthy samples. The DECs (asthma vs. healthy) of this methylation chip dataset were identified according to champ.DMP, and the results were presented in the volcano plot (Figure 2(b)). The threshold was set as adj.P.Val <10^−8^, deltaBeta <-0.05 for up-regulated DECs (*n* =121) and down-regulated DECs (*n* =20). The up-regulated and down-regulated DECs are shown in the heat map (Figure 2(c)). In the heat map, we observed that the asthma group (blue) and the healthy group (red) samples are almost separable, but some asthma samples were still mixed in the healthy group (red). Thus, the recognition ability of DECs for asthma and healthy samples still needs to be improved.

### 3.2. GO and KEGG Analyses of DECs

GO and KEGG analyses were used to understand the biological function and regulation of DECs GO results indicated that regulation of actin cytoskeleton organization and cell-substrate adhesion was enriched (Figure 3(a)). KEGG analysis showed the enrichment in shigellosis and serotonergic synapses (Figure 3(b)). The above results further confirmed that methylation played a key role in the pathogenesis of asthma. The identification of asthmatic and normal patients through a single CpGs site or multiple CpGs models is an urgent problem to be solved.

### 3.3. Differential CpGs (DECs) in the Random Forest (RF)

The above results provided a preliminary understanding of the key role of methylated CpGs in asthma. Although CpGs played an important role in differentiating asthma from healthy samples, the results are not satisfactory (Figure 2(c)). These DECs were used as the input of the random forest classifier. In order to make the error rate as small as possible, we calculated the mean error rate (err.rate), the parameter of the variable was considered to be 7, and the final neural network model incorporated 600 trees as the final model parameters to ensure that the errors were stable (Figure 4(a)). The random forest model dimension importance was obtained according to the Gini coefficient method (MeanDecreaseAccuracy and MeanDecreaseGini; Figure 4(b)). The top 10 DECs of importance were identified (cg05075579, cg20434422, cg03907390, cg00712106, cg05696969, cg22862094, cg11733958, cg00328720, cg13570892, and cg03325522). As follow-up candidates for the classification of our random forest classification results, in these DECs, cg05075579 was considered the most important, with the mean decrease of the Gini index being much higher than DECs (Table 1). The heat map (Figure 4(c)) showed that these 10 DCGs were better at clustering asthma samples together than in Figure 2(c).

### 3.4. The Construction of Artificial Neural Network Model

The random forest classifier identified the most important 10 DECs with a significant discriminative effect to distinguish between asthma and healthy samples. The artificial neural network calculated the weights of these 10 DECs, 10 input layers, seven hidden layers, and two output layers in the GSE85566 methylation expression profile and constructed a new model (Figure 5(a)). For an effective evaluation of the results of the neural network model, we chose the 10-fold cross-validation method. The data were randomly divided into a training set and validation set and used the pROC installation package to visualize the results (Figure 5(b)). In addition, we adopted the confusion matrix of the caret package to evaluate the accuracy of the neural network models (accuracy: 0.9739). Using methylation expression profiles, we developed a novel model to differentiate asthma and healthy sample classifications based on what we demonstrated above.

### 3.5. ROC Identification of the Dataset

We showed the classification of asthma and normal samples based on neural network construction. Then, we utilized two methylation datasets (GSE40576 and GSE137716) to evaluate the classification performance of our neural network model. The receiver operating characteristic curve (ROC) calculated accuracy (Figures 6(a) and 6(b)), GSE137716 dataset has AUC: 1.000, the sensitivity and specificity of 100% under the best threshold, GSE40576 dataset has AUC: 0.950, the sensitivity and specificity were 0.959 and 0.969, respectively. Comparing SVM, CART, and XGBoost machine algorithms (Table 2), the AUCs for GSE40756 are 0.825%, 0.773%, and 0.619%, respectively, and for GSE137716, AUCs are 0.938, 0.818, and 0.881, respectively. These results indicate that our neural network model had high-precision classification performance and is indicative of the classification of asthmatic patients.

## 4. Discussion

This was the first study to utilize DNA methylation-based machine learning to identify a series of asthma-related methylation loci (DECs). Interestingly, the selected methylation signatures were associated with actin cytoskeleton organization and cell-adhesion substrate, shigellosis, and serotonergic synapses, supporting the hypothesis that airway structural reorganization in asthma results from changes in DNA methylation in the epigenetic group [28, 29]. Then, ten distinct specific DECs were identified based on RF, and ANN model was built by calculating the weight coefficient of ANN. The model had high accuracy and stability (the AUC of the external validation datasets was 1 and 0.95, respectively).

Recently, due to the rapid advancement of computing power, artificial intelligence methods such as machine learning have been widely employed in medicine, including disease diagnosis and disease prognosis, thereby accelerating our understanding of various diseases. In addition, it facilitates the clinicians in patient management. Multiple studies have developed novel models to predict clinical outcomes of asthma [30–32]. In this study, we focused on the key role of epigenetics (methylation) in asthma. The asthma-related DECs were obtained through differential analysis, 10 crucial candidate DECs were identified based on the random forest classifier, and the asthma-related neural classification scores were generated by artificial neural networks. We also compared the classification efficiency of individual CpGs with the classification efficiency of the model.

We identified the methylation landscape of the methylation data (GSE85566) and obtained 142 differentially expressed CpGs. GO analysis suggested that asthma was enriched in regulation of actin cytoskeleton organization [33], cell-substrate adhesion [34], and response to nutrient levels, and KEGG results identified the potential signaling pathways, shigellosis serotonergic synapse, and yersinia infection. In addition, 10 DECs obtained through the MeanDecreaseGini importance screening of the random forest model provided a base for the construction of a neural network model. The model was highly accurate (accuracy: 0.9739), and the results were also validated with two other datasets, giving the accuracy and high classification level (AUC: 1.000 and 0.950, respectively) of this neural network. We compared our model with other currently available machine learning algorithms (SVM, CART, and XGBoost) [35, 36] and found that the diagnostic ability of the methylation machine model constructed by ANN was higher than other models.

There are several limitations to this study. First, our analysis results were based on an online database. There were more influencing factors between different datasets, which can be biased in the results. In addition, our study was limited and could not be validated in clinical patient samples. Due to the paucity of available methylation data, our dataset contains data from children's peripheral blood single cells, which may have affected the results. In future studies, we will verify our results with prospective studies in an effort to implement them in clinical practice and provide doctors with a treatment formulation source.

## 5. Conclusion

In general, our neural network model based on methylation epigenetics has a significant clinical value for the prediction of asthma, which is beneficial for early diagnosis of asthma.

## Figures and Tables

**Figure 1:** The workflow of our study.

**Figure 2:** Methylation landscape of GSE85566. (a) Heat map of the top 1000 most divergent CpGs; the gradient from dark blue to yellow represented the change in expression level. (b) Results of differential expression analysis of volcano plots (asthma vs healthy). The *X*-axis was log(deltaBeta), and the ordinate was -log10(adj.P.Val) value; DOWN (red): DECs with down-regulated expression, UP (gray): DECs with up-regulated expression, NOT (dark blue): meaningless. (c) Heat map of DECs. Dark blue to light blue means high to low expression, green represents asthma samples, red represented healthy samples, and a clustering tree aggregated similar samples together.

**Figure 3:** GO and KEGG analysis results. (a) GO analysis (including molecular function, cellular component, and biological process). (b) KEGG analysis.

**Figure 4:** (a) The effect of the number of decision trees on the error rate. The *X*-axis was the number of decision trees, and the *Y*-axis was the error rate. The increase of trees did not affect the reduction of the error rate. (b) After the variables were entered into the random forest, the top 10 DECs were listed in order of importance according to MeanDecreaseAccuracy (left) and MeanDecreaseGini (right). (c) Hierarchical clustering results of 10 DECs in GSE85566 dataset; dark colors represent high expression, light colors represent low expression, the red band above the heat map represents normal samples, and green represents asthma samples.

**Figure 5:** Neural network topology. (a) Artificial neural network visualization results for the train dataset. (b) ROC results (cg05075579, cg20434422, cg03907390, cg00712106, cg05696969, cg22862094, cg11733958, cg00328720, cg13570892, and cg03325522) analysis visualization for 10-fold cross-validation method.

**Figure 6:** Two datasets determine neural network classification efficiency. (a) ROC result of GSE137716 dataset. (b) ROC result of GSE40576. The points marked on ROC curve are the optimal threshold points, and the values in parentheses indicate sensitivity and specificity. The AUC value was the Area Under ROC Curve, *X*-axis was the specificity, and *Y*-axis was the sensitivity. The optimal threshold was marked at the inflection point, and sensitivity and specificity were listed in parentheses.

**Table 1:** MeanDecreaseGini of 10 DECs by random forest process.

CpGs	MeanDecreaseGini
cg05075579	1.427152626
cg20434422	1.421703772
cg03907390	1.395149582
cg00712106	1.355657539
cg05696969	1.099293192
cg22862094	0.981588017
cg11733958	0.933543882
cg00328720	0.897459032
cg13570892	0.880545548
cg03325522	0.879691331

DECs: differentially expressed CpGs.

**Table 2:** ROC validation results of three machine learning models (SVM, CART, and XGBoost).

Methods	GSE40576			GSE137716		
	AUC	Specificity	Sensitivity	AUC	Specificity	Sensitivity
SVM	0.825	0.845	0.804	0.938	1.000	0.875
CART	0.773	0.856	0.691	0.818	0.824	0.812
XGBoost	0.619	0.619	0.619	0.881	0.824	0.938

CART: Classification and Regression Trees; SVM: support vector machines; XGBoost: eXtreme Gradient Boosting; AUC: Area Under Curve.

## Data Availability

The data of this study were downloaded and compiled from the GEO database (https://www.ncbi.nlm.nih.gov/gds/?term=); data used to support the results of this study were obtained from the corresponding author.
